The article "Net Expression Inhibits the Growth of Pancreatic Ductal Adenocarcinoma Cell PL45 In Vitro and In Vivo" was retracted in 2024. Reasons: duplicated images; duplicated data; overlap with earlier publications; original data or images not available.

# Net Expression Inhibits the Growth of Pancreatic Ductal Adenocarcinoma Cell PL45 *In Vitro* and *In Vivo*

**DOI:** 10.1371/journal.pone.0057818

**Published:** 2013-02-28

**Authors:** Baiwen Li, Xinjian Wan, Qi Zhu, Lei Li, Yue Zeng, Duanmin Hu, Yueqin Qian, Lungen Lu, Xingpeng Wang, Xiangjun Meng

**Affiliations:** 1 Department of Gastroenterology, Shanghai First People’s Hospital, School of Medicine, Shanghai Jiaotong University, Shanghai, China; 2 Department of Gastroenterology, Ruijin Hospital, School of Medicine, Shanghai Jiaotong University, Shanghai, China; Southern Illinois University School of Medicine, United States of America

## Abstract

Pancreatic ductal adenocarcinoma has a poor prognosis due to late diagnosis and a lack of effective therapeutic options. Thus, it is important to better understand its molecular mechanisms and to develop more effective treatments for the disease. The ternary complex factor Net, which exerts its strong inhibitory function on transcription of proto-oncogene gene c-fos by forming ternary complexes with a second transcription factor, has been suspected of being involved in pancreatic cancer and other tumors biology. In this study, we found that the majority of pancreatic ductal adenocarcinoma tissues and cell lines had weak or no expression of Net, whereas significantly high level of Net expression occurred in paired adjacent normal tissues we studied. Furthermore, using *in vitro* and *in vivo* model systems, we found that overexpression of Net inhibited cell growth and survival and induced cell apoptosis in human pancreatic ductal adenocarcinoma cell PL45; the mechanisms by which Net inhibited the cell cycle progression were mainly through P21-Cyclin D1/CDK4 Pathway. Our data thus suggested that Net might play an important role in pancreatic carcinogenesis, possibly by acting as a tumor suppressor gene.

## Introduction

Pancreatic cancer is a devastating life threatening causes in the world [1], [2]. The 5-year survival rate is only 3% to 5% and has remained unchanged for the past three decades, although research progresses have been made in early diagnosis and treatments [3], [4], [5]. Therefore further understanding of its biological properties at a molecular level and identifying novel molecular targets for early diagnosis and therapeutic intervention is urgently required.

Net is a member of the ternary complex factor (TCF) subfamily of ETS-domain transcription factors [6], [7], [8]. The important function of the TCFs is to activate the immediate early genes by forming ternary complexes with a second transcription factor, a serum response factor (SRF) at serum response elements (SREs) found in the promoters of target genes [9], [10], [11]. Proto-oncogene c-fos which is upregulated rapidly upon stimulution from cells in the setting of various mitogens is fully characterized as a target of TCF. SRF has been found to be constitutively bound to the SRE in the c-fos promoter and hence be able to recruit Net [8], [12], [13], [14], [15].

The article "Net Expression Inhibits the Growth of Pancreatic Ductal Adenocarcinoma Cell PL45 In Vitro and In Vivo" was retracted in 2024. Reasons: duplicated images; duplicated data; overlap with earlier publications; original data or images not available.

Studies have suggested that the activation of the mitogen activated protein kinases (MAPKs) pathway leads to activation of Net as well as other TCFs [10], [16]. Moreover, Net is different from other TCFs by exerting its strong inhibitory function on transcription of proto-oncogene gene c-fos [17], [18], [19], [20]. C-fos, as an important component of the transcription factor activating protein 1 (AP-1), is involved in a wide variety of cellular processes, including cell proliferation, gene expression, differentiation, cell death, survival and tumorigenesis [21], [22], [23]. The transcription of c-fos is tightly controlled in normal conditions and it’s abnormal expression contributes to various phenotypical changes. Previous study suggested impaired serum inducibility of c-fos is a feature of senescent human fibroblasts [24], and its overexpression is a suggestive marker for progression of skin tumors tumorigenicity [25], [26]. However, the role of Net in pancreatic ductal adenocarcinoma is poorly understood to data.

Our previous preliminary study found that Net overexpression inhibited synthesis of the proto-oncogene c-fos in pancreatic carcinoma BxPC-3 cell [27]. In the present study, we examined the expression of Net in human pancreatic ductal adenocarcinoma and paired normal adjacent tissues, as well as in pancreatic cancer cell lines, and investigated the effect of Net expression on pancreatic ductal adenocarcinoma cell growth, proliferation and apoptosis in vitro and in vivo assays.

## Materials and Methods

### Tumour Samples and Cell Lines

The study group consisted of 21 men and 15 women with pancreatic ductal adenocarcinoma (median age 64; range 42–78 years) who underwent surgical treatment in the Department of Surgery of Shanghai First People’s Hospital and Pancreatic Disease Center of Shanghai Jiaotong University from January 2009 to March 2011. The expression of Net was evaluated on fresh pancreatic ductal adenocarcinoma tissues (PDATs) and paired normal adjacent tissues (NATs, >2 cm from tumor tissues). All the patients examined in this study had not received preoperative chemoradiation therapy. Surgical staging of tumors was performed according to the American Joint Committee on Cancer tumor-nodes metastasis system and International Union Against Cancer (2002). The clinicopathologic characteristics of patients were obtained from clinical notes and hospital computer database.

The article "Net Expression Inhibits the Growth of Pancreatic Ductal Adenocarcinoma Cell PL45 In Vitro and In Vivo" was retracted in 2024. Reasons: duplicated images; duplicated data; overlap with earlier publications; original data or images not available.

All studies were performed after written consent was obtained, according to the guidelines of the Institutional Review Board and the ethical committee of Shanghai First People’s Hospital (the approval number code: SYXK(Hu) 2009-0086). Human pancreatic ductal epithelial cell line hTERT-HPNE, pancreatic adenocarcinoma cell lines PL45, SW1990 and Panc-1 were commercially obtained from Institute of biochemistry and cell biology, SIBS, Chinese Academy of Science, and maintained in DMEM supplemented with 10% fetal bovine serum (FBS) and penicillin/streptomycin.

### Immunohistochemistry

Immunohistochemistry studies were performed according to previously described with a slight modification [28]. Briefly, formalin-fixed, paraffin- embedded tissues were de-waxed in xylene and rehydrated in graded concentration of alcohols. Following antigen retrieval and slide section blocking, tissue sections were incubated with antibodies at 4°C degree for overnight. A combined sigling nintensity and percentage of positive scoring method was used as reported previously [29]. Strong intensity staining was scored as 3, moderate as 2, weak as 1, and negative as 0. For each intensity score, the percentage of cells with that score was estimated visually. A combined weighted score consisting of the sum of the percentage of cells staining at each intensity level was calculated for each sample, e.g., a case with 70% strong staining, 10% moderate staining, and 20% weak staining would receive a score as follows: (70×3+10×2+20×1) = 250. Net immunolabeling was categorized as negative (score<30) or positive (score≥30).

### Plasmid Construction and Transfection

Net expression plasmids were constructed as previously described [28]. The full-length cDNA of Net was amplified by polymerase chain reaction (PCR). The primers were 5′-gat ctc gag atg gag agt gca atc acg ct-3′ (forward) and 5′-gag ggt acc gga ttt ctg aga gtt tga aga-3′ (reverse), which provided with the XhoI and KpnI restriction site (underlined), respectively. PCR products were cloned into pDC316 to generate a pDC316-Net plasmid. The pDC316- Net and the skeleton plasmid pBHG-fiber5/35 were subsequently co-transfected into 293 cells using Polyfect (Qiagen, Hilden, Germany) yielding the recombinant Ad5/F35-Net plasmid. Successful recombination was confirmed by observation of cytotoxicity and sequencing. The control recombinant plasmid Ad5/F35-GFP (green ﬂuorescent protein) was prepared by the same method. PL45 or hTERT-HPNE cells were transfected with Ad5/F35-Net or Ad5/F35-GFP plasmid.

### Reverse Transcription-polymerase Chain Reaction (RT-PCR)

Briefly, total RNA was extracted from cultured cells or human pancreatic tissue using the RNeasy RNA isolation kit (Qiagen, Valencia, CA) according to the manufacturer’s protocol. RNA was quantitated and PCR reactions were performed: initial denaturation at 94°C for 5 min, 35 cycles of 94°C for 40 s, 55°C for 40 s, 72°C for 90 s and an extension for 10 min at 72°C. The PCR products were electrophoresed on 1.2% agarose gels. Primers used for RT-PCR as showed in Table 1.

The article "Net Expression Inhibits the Growth of Pancreatic Ductal Adenocarcinoma Cell PL45 In Vitro and In Vivo" was retracted in 2024. Reasons: duplicated images; duplicated data; overlap with earlier publications; original data or images not available.

**Table 1:** List of primer pairs.

Net Forward	5′- acg ctg cca gta ttt cat cc -3′	387 bp
Reverse	5′-gac taa ggc tgc tcc aga aat c-3′	
P21 Forward	5′-cag ggg aca gca gag gaa ga-3′	335 bp
Reverse	5′-ggg cgg cca ggg tat gta c-3′	
P27 Forward	5′-cgg tgg acc acg aag agt ta -3′	320 bp
Reverse	5′-tct ggc tgt ccg acg gat ca -3′	
CDK2 Forward	5′-aaa ttc atg gat gcc tct gc-3′	332 bp
Reverse	5′-cga gtc acc atc tca gca aa-3′	
CDK4 Forward	5′-ccc gaa gtt ctt ctg cat tc-3′	313 bp
Reverse	5′-agg cag aga ttc gct tgt gt-3′	
Cyclin D_1_ Forward	5′-att gtg atc agg tgt cca ca- 3′	380 bp
Reverse	5′-tac ttg acg gcc acg gac at-3′	
Cyclin E Forward	5′-act caa cgt gca agc ctc gg-3′	400 bp
Reverse	5′-gaa caa gct cca tct gtc ac-3′	
c-Fos Forward	5′- tgt caa cgc gca gga ctt ct -3′	443 bp
Reverse	5′- cct tct cct tca gca ggt tg -3′	
c-Jun Forward	5′-agc tgg aga gaa tcg ccc ggc tg-3′	356 bp
Reverse	5′-cca agt cct tcc cac tcg tgc aca ct-3′	
β-actin Forward	5′-tga cgg ggt cac cca cac tgt gcc cta cta -3′	658 bp
Reverse	5′-cta gaa gca ttt gcg gtg gac gat gga ggg	

### Western Blot

Cells at 70∼80% confluency were washed with PBS and then lysised on ice for 20 min. The protein was quantified using a BCA protein assay kit (Pierce, Rockford, Illinois, USA). Cell lysate (30 µg) was separated on 10% SDS-PAGE gel and transferred to polyvinylidene ﬂuoride (PVDF) membrane using a Bio-Rad transfer system and then visualized with ECL detection system (Amersham Pharmacia Biotech, Piscataway, NJ, USA).

### Cell Viability Assessment

Cell viability was assessed via MTT test as previously described [27]. The absorbance of the samples was measured using a microplate reader at 570 nm.

### Cell Cycle Analysis

Cells seeded in six well plates were harvested when they are 70–80% confluent, and then washed twice with PBS. The cells were resuspended in 0.5 ml of PBS and fixed with 70% ethanol. Cells were resuspended in 0.2 mg/ml of propidium iodide (PI) containing 0.1 mg/ml RNase A, and incubated in the dark for 30 min at room temperature before analyzed on FACScan flow cytometer. The percentage of cells in different phases of the cell cycle was assayed using a ModFit 5.2 computer program.

### Colony Formation Assay

Soft agar colony formation assay was used to assess the anchorage-independent growth ability of cells as previously described [27]. Agarose (0.6%) in DMEM was casted on six-well plates. Cells (1×10^3^ cells/well) were mixed with 0.3% agarose in DMEM containing 10% FBS at 37°C and seeded over the agarose. Colonies larger than 50 µm were counted at 15 days after plating.

The article "Net Expression Inhibits the Growth of Pancreatic Ductal Adenocarcinoma Cell PL45 In Vitro and In Vivo" was retracted in 2024. Reasons: duplicated images; duplicated data; overlap with earlier publications; original data or images not available.

### Propidium Iodide Staining

Brieﬂy, cells (1×10^6^ cells/mL) cultured in 24-well ﬂat bottom plates were harvested, washed with cold phosphate-buffered saline and resuspended in PBS containing propidium iodide. After 20 minutes incubation, cells were examined with fluorescence microscope at emission 636 nm.

### Ultrastructural Analysis

Cell monolayers were washed, fixed with 2.5% glutaraldehyde in 0.1 M phosphate buffer for 15 min, gently scraped, and centrifuged at 1200 rpm. Cell pellets were further fixed by glutaraldehyde for 1 h. All specimens were post fixed in OsO4, alcohol dehydrated, and embedded in araldite, as previously described [30]. Thin sections were stained with uranyl acetate and lead citrate and analyzed with a Philips CM10 electron microscope.

### Nude Mouse Xenograft Model

To examine the effects of Net gene overexpression on tumour growth in vivo, xenograft model of nude mice with pancreatic cancer was established. Balb/c nude mice were maintained under specific pathogen-free condition in Shanghai Experimental Animals Centre of Chinese Academy of Sciences. All protocols and procedures in animal study were approved by the Ethics Committee of Shanghai First People’s Hospital and following current China Guidelines. PL45 cells (1×10^7^ suspended in 100 µl of PBS) were subcutaneously injected into the hind flank of 5–6 weeks old Balb/c nude mouse. As the tumour grew larger, it was resected, slashed into small even slices in aseptic condition, and replanted into the hind flanks of Balb/c nude mice. Tumours were implanted subcutaneously in mice to more than passage three. When the tumours were palpable, animals were randomly divided into three groups (8 in each group): (a) control group, animals were injected directly into the tumours with PBS every third day. (b) Ad5/F35-GFP group, animals were injected directly into the tumours with 1×10^8^ pfu (plaque-forming units) Ad5/F35-GFP every third day; and (c) Ad5/F35-Net group, animals were injected directly into the tumours with 1×10^8^ pfu adenovirus containing Net gene (Ad5/F35-Net) every third day. Body weight and volume of xenografts were measured in a blinded fashion using callipers every third day during the three weeks treatment period. Tumour volume (V) was estimated from tumour length (l) and width (w) using the formula V = lw2 π/6. Total mRNA was prepared from every group tumours and RT-PCR analyses were performed as described previously. Tunel assay and PCNA staining were used to evaluate cell proliferation and apoptosis according to the procedure previously described [28]. Positively stained cells were sorted as the percentage of total tumour cells in five high resolution fields.

The article "Net Expression Inhibits the Growth of Pancreatic Ductal Adenocarcinoma Cell PL45 In Vitro and In Vivo" was retracted in 2024. Reasons: duplicated images; duplicated data; overlap with earlier publications; original data or images not available.

### Statistical Analysis

Results are expressed as the mean ± S.E.M. Each experiment was repeated at least three times. Statistical significance of difference between test groups was assessed by one-way ANOVA followed by Scheffe’s test (post hoc). The Kruskal-Wallis or Mann-Whitney U-tests was used to compare the difference of Net expression in age, sex, tumor size, tumor classification, localization and pathological stage. All statistical analyses were performed using SPSS 16.0 software. Statistical significance was defined at p<0.05.

## Results

### Down-regulation of Net in Pancreatic Carcinoma

36 cases of human pancreatic ductal adenocarcinoma tissues and matched adjacent normal tissue samples were examined for the expression of Net by immunohistochemistry. The neoplastic cells of low proportions (16.7%) of pancreatic carcinoma tissues expressed Net (6 cases in 36 cases), which was highly expressed on majority (88.9%) of paired normal adjacent tissues (32 cases in 36 cases). On the contrary, high expression of c-fos and Ras were detected in pancreatic carcinoma tissues compairing with low expression in peritumor tissues. While both Net and c-fos were mainly located in nucleus, Ras was located in cytoplasmic, the brown-yellowish staining indicate the positive cells (Fig. 1A). Semi-quantitative RT-PCR and Western blot were used to evaluate the changes of Net expression in both mRNA and protein levels in pancreatic carcinoma tissues. The results showed that Net expression was down regulated both at mRNA and protein levels in pancreatic carcinoma tissue in relative to that in peritumor tissues (Fig. 1B). Pancreatic carcinoma cell lines PL45, SW1990, PANC-1 and human pancreatic cell line hTERT-HPNE were employed and similar results were obtained, expression of Net mRNA and protein in pancreatic carcinoma cell lines (especially in PL45 cell line) were significantly lower than that in human pancreatic cell line (Fig. 1C).

**Figure 1:** Net is down-regulated in pancreatic ductal adenocarcinoma. (A) Immunohistochemical analysis of Net, c-fos and Ras expression in pancreatic ductal adenocarcinoma tissues (top row) and matched adjacent normal tissue samples (bottom row). a and b is H&E staining with low resolution (×100); c, d denote the expression of Net representative with high resolution (×200); e, f denote the expression of c-fos representative with high resolution (×200); g, h denote the expression of Ras representative with high resolution (×200). (B) Expression of Net was examined at mRNA and protein levels using RT-PCR and western blotting on human pancreatic ductal adenocarcinoma tissues (T) and matched adjacent normal tissue samples (N) (presentive 5 cases of 36). (C) Expression of Net was examined at mRNA and protein levels using RT-PCR and western blotting in pancreatic cancer cell lines (SW1990, PANC-1 and PL45) and human pancreatic cell hTERT-HPNE. PDAT, pancreatic ductal adenocarcinoma tissues; NAT, normal adjacent tissue.

The article "Net Expression Inhibits the Growth of Pancreatic Ductal Adenocarcinoma Cell PL45 In Vitro and In Vivo" was retracted in 2024. Reasons: duplicated images; duplicated data; overlap with earlier publications; original data or images not available.

The correlation of Net Immunohistochemistry score with a variety of clinicopathologic factors was evaluated with Kruskal-Wallis or Mann-Whitney U-tests in 36 patients with pancreatic ductal adenocarcinoma. Patients with weak or no expression of Net appeared to have high level of CA19-9 and node involvement (P<0.01). However, Net expression was not correlated with age, gender, localization of tumor, or differentiation. Although there was difference in tumour classification and clinical staging between patients with high expression of Net and patients with weak or no expression of Net, no statistical significance was observed. The few case number of patients may account for that.(As shown in Table 2).

**Table 2:** Relationship between Net IHC score and clinicopathologic factors in 36 patients with pancreatic ductal adenocarcinoma.

Parameter	n	Net IHC score		
		<30	≥30	*P* Value^a^
Age				1.0
≤60	14	12	2	
>60	22	18	4	
Gender				0.655
Male	21	17	4	
Female	15	13	2	
Localization				1.0
Head	20	17	3	
Other	16	13	3	
CA19-9 (U/L)				0.014
≤100	8	4	4	
>100	28	26	2	
Size (cm)				0.662
≤3	19	15	4	
>3	17	15	2	
Differentiation				0.643
Well/moderate	25	20	5	
Poor	11	10	1	
Tumour classification^b^				0.385
T1/T2	23	18	5	
T3/T4	13	12	1	
Nodal status				0.001
N0	13	7	6	
N1	23	23	0	
Pathological stage				0.304
I/II	26	20	6	
III/IV	9	9	0	

a Kruskal-Wallis test and Mann-Whitney U-test.

b Tumor classification was made according to International Union Against Cancer (2002).

### Overexpression of Net Inhibits the Growth and Proliferation of Pancreatic Ductal Adenocarcinoma Cell PL45

PL45 cells that expressed low level of Net were transfected with adenovirus vector that encodes Net (Ad5/F35-Net) to make cells that expressed high level of Net. Cells were examined for growth and proliferation following transfection. Results indicated that the growth and proliferation ability of PL45 cell transfected with Ad5/F35-Net was significantly inhibited in relative to PL45 cells without transfection (control) or transfected with control vector Ad5/F35-GFP (P<0.01) (Fig. 2A, 2B); The number of colony formation was significantly reduced as well in cells transfected with Ad5/F35-Net (Fig. 2C). All those results suggested that Net play a role in inhibiting the proliferation of pancreatic ductal adenocarcinoma cell PL45. Moreover, cell cycle results revealed that most of PL45 cells transfected with Ad5/F35-Net were delayed in G0/G1 phase (59.96±8.54%) after 48 hours transfection in comparing with cells transfected with Ad5/F35-GFP (44.45±4.75%) or control PL45 cells (44.45±4.75%) respectively. The cells in S phase (26.57±5.64%) were significantly lower in cells transfected with Ad5/F35-Net than that in cells transfected with Ad5/F35-GFP (45.73±4.68%) or control cells (45.84±5.36%) (Fig. 2D) (P<0.01), which suggested that the overexpression of Net can delay pancreatic ductal adenocarcinoma cell PL45 at G0/G1 phase.

The article "Net Expression Inhibits the Growth of Pancreatic Ductal Adenocarcinoma Cell PL45 In Vitro and In Vivo" was retracted in 2024. Reasons: duplicated images; duplicated data; overlap with earlier publications; original data or images not available.

**Figure 2:** Net inhibited growth and proliferation in pancreatic ductal adenocarcinoma cell PL45. (A) Growth of PL45 cells transfected with or without Ad5/F35-Net was measured by MTT assay. (B)The growth curve of PL45 cells transfected with or without Ad5/F35-Net was obtained by counting cell numbers per well on each day. (C) Colony formation assay was performed using PL45 cells transfected with or without Ad5/F35-Net after 48 h. (D) Cell cycle of PL45 cells transfected with or without Ad5/F35-Net was evaluated. (E) Cell cycle related genes were examined at mRNA and protein levels 48 hours after Ad5/F35-Net transfection. *p<0.05, **p<0.01.

### Net Inhibits Cell Cycle Progression through p21-Cyclin D_1_/CDK_4_ Pathway

To further investigate the mechanisms by which Net inhibits pancreatic ductal adenocarcinoma cell PL45 proliferation, several cell cycle associated genes (p21, p27, CDK2, CDK4, Cyclin D_1_, Cyclin E,c-Jun, and etc.) were evaluated at mRNA and protein levels 48 hours after Ad5/F35-Net infection. The results showed that overexpression of Net inhibited c-fos expression in both mRNA and protein levels. While the expression of p21 was up-regulated by overexpression of Net, the expression of Cyclin D_1_ and CDK4 were down-regulated following transfection of Net. No obvious changes were observed for the expression of p27, CDK2, Cyclin E and c-Jun before and after transfection (Fig. 2E).

### Net Expression Induces the Apoptosis of Pancreatic Ductal Adenocarcinoma Cell PL45

The apoptosis of PL45 cell was evaluated by AnnexinV/PI staining method after 48 hours of Ad5/F35-Net transfection. The early period apoptosis potential of control cells, cells transfected with Ad5/F35-GFP or Ad5/F35-Net group was 5.81±1.6%, 5.90%±1.3 and 46.32±8.1% respectively. The differences between Ad5/F35-Net and control or Ad5/F35-GFP group were significant (P<0.01), while there was no significant difference between control and Ad5/F35-GFP group (P>0.05). The enhanced apoptotic ability of cell transfected with Ad5/F35-Net occurred in the early stage but not in the late stage, there were no statistical difference in the late stage of apoptosis among three groups (32.32±4.1%, 32.61%±4.4 and 34.64±4.7%, respectively. Fig. 3A, 3B). Ultrastructures of cells were observed by TEM (Transmission Electron Microscope) after transfection. We found that PL45 cell transfected with Ad5/F35-Net demonstrated concentrated phenomena of cytoplasm, density increasing, nuclear chromatin margination, karyopyknosis and karyorrhexis, apoptotic body formation, while no obvious changes was observed in neither control group or Ad5/F35-GFP group (Fig. 3C). Our results suggested that overexpression of Net induced the apoptosis of PL45 cell.

The article "Net Expression Inhibits the Growth of Pancreatic Ductal Adenocarcinoma Cell PL45 In Vitro and In Vivo" was retracted in 2024. Reasons: duplicated images; duplicated data; overlap with earlier publications; original data or images not available.

**Figure 3:** Net induces the apoptosis in pancreatic ductal carcinoma cell PL45. (A) Cell apoptosis was examined in PL45 cells after 48 hours of Ad5/F35-Net transfection using AnnexinV/PI method. (B) The rates of early and late apoptosis were evaluated after 48 hours of Ad5/F35-Net transfection. (C) Ultrastructures of cells were observed by transmission electron microscope. Concentrated phenomena of cytoplasm, karyopyknosis, karyorrhexis and apoptotic body formation were detected in PL45 cell transfected with Ad5/F35-Net, no obvious changes was observed in control group and Ad5/F35-GFP group. Black arrow indicated karyopyknosis andkaryorrhexis. *p<0.05, **p<0.01.

### Overexpression of Net Inhibits Growth of Transplanted Pancreatic Carcinoma in Nude Mice

To examine the effect of Net on human pancreatic carcinoma growth in *in vivo*, xenograft model of human pancreatic carcinoma in nude mice was established. The average tumor size and weight were significantly reduced in nude mice injected with PL45 cells transfected with Ad5/F35-Net 21 days later compared with that in mice injected with control cells or cells transfected with Ad5/F35-GFP (P<0.05, Fig. 4A, 4B) indicating that the overexpression of Net inhibits the growth of pancreatic carcinoma in mice. RT-PCR and Immunohistochemistry assay showed that over-expression of Net resulted in decreased c-fos expression and increased P21 expression both in mRNA and protein levels in xenograft tissues (Fig. 4C, 4D). PCNA stain results demonstrated that PCNA labeling index was significant lower in xenograft tissues with cells transfected with Ad5/F35-Net (42.9%) than that with control cells (74.1%) or cells transfected with Ad5/F35-GFP (68.7%) (P<0.01, Fig. 4E). On the other hand, apoptotic cells detected by TUNEL assay showed that the apoptotic index of xenograft tissues with cells transfected with Ad5/F35-Net(18.2%) was significant higher than that with control cells (5.4%) or cells transfected with Ad5/F35-GFP group (4.9%) (P<0.01, Fig. 4E), which suggested that Net had the ability to prohibit pancreatic carcinoma xenograft growth in nude mice through inhibiting proliferation and inducing cell apoptosis.

The article "Net Expression Inhibits the Growth of Pancreatic Ductal Adenocarcinoma Cell PL45 In Vitro and In Vivo" was retracted in 2024. Reasons: duplicated images; duplicated data; overlap with earlier publications; original data or images not available.

**Figure 4:** The effects of Net expression on tumor growth in vivo. (A) Tumor size was measured every three days interval in each group. (B) Weight of dissectable xenograft tumors was measured in each group. (C) Expression of Net, c-fos and P21 in mRNA levels in xenograft tissues. (D) Representative H&E staining, histological staining of Net, c-fos and P21, PCNA staining and TUNEL assay in xenogrft tissues. (E) Index of PCNA and apoptosis were accounted in xenograft tumour tissues. *p<0.05, **p<0.01.

## Discussion

Net, an important transcription regulator and downstream target of Ras-MAPKs pathway, has the ability to regulate protooncogene c-fos transcription by forming a ternary complex on the promoter of target gene and eventually affect cell proliferation and differentiation [21], [23]. Low expression of Net has been reported in some carcinoma cells such as cervical cancer and overexpression of Net could inhibit the growth of cervical carcinoma cell [31], but the mechanism is still unknown. It was not known whether other tumors (including pancreatic carcinoma) expressed Net and its fnctional significance. In this study, human pancreatic ductal adenocarcinoma tissues and pancreatic adenocarcinoma cell lines were examined for the expression of Net using immunohistochemistry, RT-PCR, and Western blot. Results showed that pancreatic ductal adenocarcinoma tissues and cell lines expressed relatively low level of Net and an inverse correlation was found between the expression of Net and c-fos or Ras in the tissues and cells, which was in agreement with our previous reports and implied that Net could inhibit the expression of c-fos [27]. The clinicopathologic factors analysis revealed low level of Net expression was correlated with high level of CA19-9 and node involvement. These results suggested that lack of Net expression might have biological and clinical importance on pancreatic ductal adenocarcinoma.

Genetically manipulating the expression of Net provides a useful tool to examine the impact of Net on cancer growth. Previous studies suggested that Net could inhibit the growth of pancreatic cancer cell BxPC-3 transfected with Net [27]. In present study, adenovirus vector Ad5/F35-Net was constructed and transfected into human pancreatic ductal adenocarcinoma cell PL45. We found that overexpression of Net could inhibit the growth and colony formation of pancreatic carcinoma and induced delayed G0/G1 phase. TEM examination showed that stable expression of Net promoted apoptosis of PL45. Ultrastructure damage was found in Net overexpression pancreatic carcinoma cells, which was characterized by forming apoptotic bodies. Overexpressing of Net induced apoptosis. We hence postulated that Net might inhibit the proliferation of pancreatic ductal adenocarcinoma cells and promote apoptosis, and eventually preventing the development of pancreatic cancer. To confirm our hypothesis, xenograft model of the human pancreatic carcinoma in nude mice were used to study the effects of Net expression on tumor development, results also indicated that Net overexpression inhibits the growth of xenograft pancreatic carcinoma with down-regulation of c-fos and up-regulation of P21 expression in vivo. In addition, we also noticed that decreased PCNA index and increased apoptotic index by overexpression of Net. These results suggested that Net has the inhibitory effects on pancreatic tumor cell growth and development in vitro and in vivo.

The article "Net Expression Inhibits the Growth of Pancreatic Ductal Adenocarcinoma Cell PL45 In Vitro and In Vivo" was retracted in 2024. Reasons: duplicated images; duplicated data; overlap with earlier publications; original data or images not available.

Given the fact that progression of cell cycle from G1 to S phase in mammalian cell is controlled by the cyclin A, cyclin D, and cyclin E, which bind to and activate different kinases in G1, such as CDK4, CDK6 and CDK2. Activation of cyclin D1/CDK4, cyclin D1/CDK6 and cyclin E/CDK2 complex is required for cell transition from G1 to S phase. Cyclin D1/CDK4 or cyclin D1/CDK6 complex are involved in early G1 phase and cyclin E/CDK2 complex is involved in mid-to-late G1 stage. Former studies showed that cyclin-CDK complexes were associated with cyclin kinase inhibitors (ckis), that bind and inactivate cyclin-CDK complexes [32],[33],[34]. P21 and p27 are proteins that bind CDK2- and CDK4-cyclin complexes, and p21 is a major inhibitor during the G1 phase of the cell cycle [33],[35],[36]. Net is activated through phosphorylation by mitogen activated protein kinases (MAPKs) [32], The phosphorylated Net in turn binds to the response element of c-fos gene promoter, leading to c-fos transcription. c-Fos protein dimerizes with c-Jun protein to form AP-1 complex, thereby regulating various target genes involved in cell proliferation and cell cycle progression [37], [38]. AP-1 complex has been shown to transactivate cyclin D1 gene and stimulate G1 to S progression [26], [39]. To understand the molecular mechanisms by which Net inhibits cell cycle progression, multiple genes associated with cell cycle such as Cyclin D, Cyclin E, CDK2, CDK4, P21, P27, c-fos and c-Jun were examined by RT-PCR and Western Blot, we found that P21 expression was increased in PL45 cells following transfection of Ad5/F35-Net, while Cyclin D_1_ and CDK4 expression was decreased, expression of CDK2 showed no obvious change. All these suggested that the effect of Net on delaying cell cycle might through the pathway of P21-Cyclin D_1_/CDK4. Since AP-1 is a heterodimer constituted by c-fos and c-Jun, c-Jun expression was also checked. However, no obvious change of c-Jun was found due to the expression of Net, suggesting that down-stream transcription regulation of Net was probably modulated by c-fos pathway but not c-Jun pathway.

The article "Net Expression Inhibits the Growth of Pancreatic Ductal Adenocarcinoma Cell PL45 In Vitro and In Vivo" was retracted in 2024. Reasons: duplicated images; duplicated data; overlap with earlier publications; original data or images not available.

In summary, the present results suggested that Net has the potential to inhibit the growth of human pancreatic ductal adenocarcinoma cell PL45 and induce cellular apoptosis in vitro and in vivo. The inhibitory mechanism is presumably by inhibiting the expression of c-fos, subsequently inactivating the transcription activity of AP-1, followed by activating of p21 to antagonize the effects of Cyclin D/CDK4 on cell cycle progression, and ultimately leading to cell death. On the contrary, intra or extracellular signals through Ras-MAPKs pathway induce phosphorylation of Net, which results in downregulating Net expression and disabling inhibitory ability of Net on c-fos transcription, thus accelerating cell cycle progression and promoting cell proliferation (the possible regulatory model as showed in Fig. 5). Further studies will be pursued to fully characterized the mechanism.

**Figure 5:** The possible regulatory model of effect of Net on pancreatic ductal adenocarcinoma. Net inhibits the growth of pancreatic ductal adenocarcinoma cell by inhibiting the expression of c-fos, subsequently inactivating the transcription activity of AP-1, followed by activation of p21 to antagonize the effects of Cyclin D/CDK4 on cell cycle progression, and ultimately leading to cell death. On the contrary, phosphorylation of Net is activated by intra or extracellular stimulation signals through Ras-MAPKs pathway, which results in downregulation of Net expression and lack of inhibitory ability on c-fos transcription, thus promoting cell proliferation.
